The article "Early Detection and Diagnosis of Chronic Kidney Disease Based on Selected Predominant Features" was retracted in 2023. Reasons: signs of a paper mill; compromised peer review; unreliable results or conclusions.

# Early Detection and Diagnosis of Chronic Kidney Disease Based on Selected Predominant Features

**DOI:** 10.1155/2023/3553216

**Published:** 2023-01-30

**Authors:** Zahid Ullah, Mona Jamjoom

**Affiliations:** ^1^Department of Information Systems, Faculty of Computing and Information Technology, King Abdulaziz University, Jeddah, Saudi Arabia; ^2^Department of Computer Sciences, College of Computer and Information Sciences, Princess Nourah Bint Abdulrahman University, Riyadh, Saudi Arabia

## Abstract

In numerous perilous cases, a quick medical decision is needed for the early detection of chronic diseases to avoid austere consequences that may be fatal. Chronic kidney disease (CKD) is a prevalent disease that presents a variety of challenges, including soaring costs for intervention, urgency, and, more importantly, difficulty in early detection of the disease. The current study carries out a prediction-based method that helps in detecting and diagnosing CKD patients which enables a fast and accurate decision-making process at the early stage. A combination of preprocessing and feature selection methods was developed; additionally, several prediction models, such as K-nearest neighbor (KNN), support vector machine (SVM), random forest (RF), and bagging, were trained based on the processed dataset. The performance evaluation shows higher reliability of all models in terms of accuracy, precision, sensitivity, F-measure, specificity, and area under the curve (AUC) score. Specifically, KNN outperformed with an accuracy of 99.50%, sensitivity of 99.2%, precision of 100%, specificity of 98.7%, and F-measure and AUC score of 99.6%. The experimental results of KNN show the best fitted model compared to the existing state-of-the-art methods. Moreover, the reduced feature set proves that just a few clinical tests are enough to detect CKD, resulting in diagnosis cost reduction.

## 1. Introduction

In the human body, the kidneys, two bean-shaped organs positioned under the ribs, play the important role of filtering wastes and toxic bodies from the blood. Chronic kidney disease (CKD) is a condition in which the human kidneys are damaged and unable to filter the blood in a proper way [1]. It is a nontransmissible disease that causes mortality of large numbers worldwide [2, 3] and is very expensive to properly detect and diagnose [3]. CKD is commonly destructive, expensive, onerous, and often risky; therefore, CKD patients often reach its chronic stages, especially in countries with limited resources [4]. Furthermore, CKD is a silent killer due to the lack of physical symptoms at the initial stage, but a steady loss of glomerular filtration rate (GFR) occurs over a period of time longer than three months [5]. The study of Bikbov et al. [2] reported that in 2016, the CKD-affected individuals reached above 752 million of which more than 335 million are males and 417 million are females. A total CKD-affected population exceeding 600 million in 112 countries cannot afford renal transplantation which leads to an annual mortality rate of over 1 million people due to kidney failure [6]. Similarly, due to CKD, the worldwide death rate of patients of any age increased by over 41% from 1990 to 2017, resulting in the mortality of 1.2 million in 2017 only [7].

CKD is a fatal disease if left undetected as it leads to renal failure, in the worst cases. However, the early diagnosis of CDK can significantly reduce the mortality rate. Moreover, if CKD is predicted early and correctly, it results in an increased probability of successful treatment and prolongs the patient's life [8]. The stages of CKD are primarily based on the estimated GFR (eGFR) which is based on creatinine level, age, and race [9]. In this regard, an efficient prediction is more useful as it can save the lives of thousands of patients and prevent negative outcomes. ML techniques play a vital role to provide fast predictions depending on historical medical data; however, it has been challenging to determine which prediction model is more accurate in a short period [10]. The advances in ML, in addition to predictive analytics, provide promising results which in turn prove the capability of prediction in CKD and beyond [11]. The utilization of ML methods in nephrology enables the building of ML models to better detect the at-risk patients of CKD and better enhance their decision-making process, especially in primary care settings [12].

This paper is an attempt to assist physicians in detecting and diagnosing CKD patients using ML techniques, simultaneously reducing the cost of diagnosing through limiting the clinical tests which will be ideal for countries with limited resources. We have trained KNN, SVM, RF, and bagging on a dataset taken from the UCI repository. The dataset was preprocessed which entailed missing value imputation, feature selection, and features normalization. The socioeconomic aim of this paper is to lessen clinical expenses and accommodate early treatment plans by achieving accurate prediction using simple and inexpensive clinical tests.

The remainder of this study is organized as follows: Section 2 discusses the previous work, while details of the methods used are discussed in Section 3, followed by results and discussion in Section 4; finally, Section 5 concludes this study.

## 2. Literature Review

Previous works related to detecting and diagnosing CKD were researched using various scholarly databases: Google Scholar, ScienceDirect, ResearchGate, Wiley Online Library, SpringerLink, IEEE Xplore, ACM Digital Library, and many more. The primary keywords used included “detection of CKD using machine learning,” “prediction models for CKD data,” and “ML methods used for detecting CKD.” In the literature, there are numerous studies available that utilized CKD data and built prediction models depending on the type of data analyzed. This study will discuss some of the related works available in the literature retrieved from the above data sources. The study of Ghosh et al. [10] attempted to achieve a fast and accurate prediction model to detect symptoms at an early stage in order to save the lives of patients suffering from CKD. They trained several ML models: SVM, AB, LDA, and GB, with CKD dataset (i.e., different from our study) and concluded that a GB model achieved the highest accuracy rate of 99.8%, followed by SVM (99.5%), and finally AB and LDA (97.91%). Moreover, the study of Gudeti et al. [13] aimed to diagnose CKD at an early stage, and as a result, they trained SVM, KNN, and LR models, which achieved accuracy rates of 99.25%, 78.75%, and 77.25%, respectively. In the study by Rashed-Al-Mahfuz et al. [3], a reduced dataset was selected based on different clinical tests and feature significance. Afterward, several ML models were built. According to their investigations, RF outperformed in terms of accuracy; therefore, the researchers concluded that RF and the reduced dataset could be used to potentially reduce the diagnosis cost and enable better decision making for early treatment plans. Similarly, Abdullah et al. [14] presented a study on the performance comparison of ML algorithms for classifying CKD. First, they selected the relevant features using five different methods for feature selection and then applied several ML algorithms (i.e., RF, SVM, NB, and LR) to evaluate the datasets. They found that the performance of the RF classifier with RF feature selection was the best among other models in terms of accuracy, sensitivity, and precision which were 98.82%, 98.04%, and 100%, respectively.

The authors of [11] investigated the capability of various ML methods to identify the early prediction of CKD. For this, they used predictive analytics in which they first examined the correlation between data features and the target class feature, resulting in 30% of data reduction which was used for predicting CKD. Furthermore, they concluded that the prediction models performed well in terms of precision, recall, and AUC. Specifically, the accuracy rate was 95.6%, 95%, 98.1%, and 98.1% for RPART, SVM, LR, and MLP in order. Likewise, Anantha Padmanaban and Parthiban [15] attempted to utilize DT and NB methods for predicting early detection of CKD for diabetic patients and concluded that the performance of DT was promising and resulted in a 91% accuracy rate while NB achieved 86% accuracy. Additionally, the authors of [16] utilized several statistical methods and association rules to help medical practitioners take precautionary measures. Moreover, several common ML methods were used for advanced prediction of CKD, and it was concluded that the combination of DT and Adam-deep learning can be more contributive to saving human lives with 97.34% accuracy. The authors of [1] trained seven ML models based on the CKD dataset and assessed them with several distinctive evaluation measures: MAE, RMSE, RAE, RRSE, recall, precision, F-measure, and accuracy. Their investigations found that Composite Hypercube on Iterated Random Projection (CHIRP) outperformed in terms of lessening error rates and increasing accuracy. The reported accuracy for CHIRP was 99.75%. Another study [8] utilized the CKD dataset and predicted the kidney diseases after selecting the most relevant features using ML methods. They have trained DT, RF, and LR based on the reduced dataset and concluded that LR was the highly reliable model in terms of actuary and recall, while DT outperformed in terms of precision. The models DT, RF, and LR attained an accuracy rate of 98.48%, 94.16%, and 99.24%, correspondingly. The authors in [17] made an attempt, using several statistical tools for feature selection and reduced the dataset to the most relevant small features. Based on the reduced data, LR, SVM, RF, and GB models were trained, and resulting accuracies were 98.75%, 97.5%, 98.5, and 99%, respectively. In addition, they found that GB was more reliable in terms of F-measure. On further investigation, hemoglobin was found to be the highly correlated predictor on both RF and GB methods. Moreover, they also concluded that with the implementation of their models, CKD can be detected with 3 simple tests priced as low as $26.75.

## 3. Materials and Methods

In this section, a detailed methodology used in this study is discussed. A complete process of data analysis for detecting and diagnosing CKD was implemented using Weka software [18]. Weka features numerous ML methods and techniques for training and testing the models and providing predictions based on the data provided for unseen cases [19–21]. The step-by-step methods used in this study are discussed in the following sections.

### 3.1. Data Collection

The dataset used in this study to detect and diagnose chronic kidney diseases was harvested from the publicly available UCI Machine Learning Repository [22]. The dataset originally contained 400 records of 24 features and a class feature. Among the 24 features, 14 are nominal and 11 are numeric while the class feature determines whether or not the case is CKD. The details of the dataset are shown in Figure 1.

### 3.2. Data Preprocessing

There were numerous missing values in the collected data. In ML and predictive analytics, decisions are always based on historical data [23]. Therefore, the data must be clean of noise and complete [24, 25] in order to have reliable predictions for future decision making [26, 27].

In this study, the categorical data were processed using a filter method converting nominal attributes to numerical attributes. The filter method used for converting nominal attributes to numerical attributes is referred to as “OrdinalToNumeric” which is an attribute filter that transforms ordinal nominal features into numeric ones [28]. The imputation of the missing values was performed using an ML method referring to DT-based missing value imputation (DMI) that uses the combination of DT and expectation-maximization (EM) algorithms for imputing missing values. In this method, EMI is applied on every leaf of a DT that utilizes the correlations of feature values of data for imputation. This approach is more advantageous in terms of high correlation within a leaf than within the entire dataset. Thus, the application of EMI yields potentially better imputation outcomes for those records belonging to a leaf compared to the whole dataset [29].

### 3.3. Feature Selection

In predictive analytics, feature selection is conducted to choose the most relevant features in a dataset and omit those features that have lower predictive accuracy in the model. In fact, this is a significant procedure for discovering accurate models. Therefore, ML provides several methods for feature selection to accomplish effectual data reduction for accurate prediction models [30], such as filter, wrapper, embedded, and hybrid methods [31, 32]. In this study, feature selection was performed using the filter method. The filter method offers optimal approaches, especially in providing an explainable feature selection process and avoiding the creation of less explainable features [33]. The mechanism used in these methods assigns a relevance score to each feature in the dataset, and based on the generated scores, the features are ranked [34]. Then, features with high rank are selected, and low rank features are then excluded [35]. The finalized dataset for detecting and diagnosing CKD after feature selection is shown in Figure 2.

### 3.4. Prediction Models

The use of artificial intelligence, in general, and machine learning, in particular, has made it possible to organize and structure the unorganized and unstructured data in such manner to have an essential part of a business decision support system. The extraction of meaningful insights from raw data and the subsequent construction of prediction models based on those data are advantages of ML methods which are broadly used in the healthcare industry for predictive analytics and decision support systems that help medical practitioners in diagnosing several diseases, among other clinical practices. There are numerous studies available in the literature that utilized ML techniques for predicting CKD. The commonly used methods in the literature are DT, KNN, RF, SVM, and NB. In this study, the ML methods used for detecting and diagnosing CKD are discussed in the following sections.

#### 3.4.1. K-Nearest Neighbor (KNN)

In this method, the data samples are labeled with distinct classes which are used for learning to label the new samples. This classification is typically based on the labels that are most closer to those of its neighbors, as well as the mainstream of votes cast. Thus, the labels of the closest neighbors are the labels of the new data points. Moreover, in this method, K is a measure for screening the nearest neighbors [36, 37].

#### 3.4.2. Support Vector Machine (SVM)

SVM is a predictive ML method that is used to find the hyperplane that amplifies the separation between classes. A hyperplane sorts the values and separates positive values from negative with maximum margin. In this method, the instances are represented as points in space. The points that are near to the maximum margin are the support vectors [38].

#### 3.4.3. Random Forest (RF)

This method utilizes the entered data and creates multitudes of DTs at the time of training and delivers a mean prediction of each tree [5]. In RF, the classification is conducted through nominating different randomized DTs on the final score where each DT is randomized based on a bootstrap resampling method with arbitrary feature selection. This practice is repeated throughout the forest for all trees based on various bootstrap data, and the new samples are labeled to the class having the majority of votes [39].

#### 3.4.4. Bagging

Bagging (bootstrap aggregation) is an ensemble method in which a training set is used to create a repeated sample based on simple random sampling with replacement whereby a weak classifier is trained for each bootstrap. The prediction of class labels on testing data is based on these trained classifiers, and thus a class with the highest votes wins [37].

### 3.5. Performance Evaluation Method

Performance evaluation of the prediction models trained can be performed in different methods such as providing the testing set as training, specifying an independent test set, specifying a percentage split, and cross-validation with the number of folds. According to [40], cross-validation is deemed to be the most reliable evaluation method. Therefore, this study has used the practice of cross-validation of 10 folds [41] for each model trained. In 10-foldcross-validation, the training dataset is subdivided into 10 splits, and each split is utilized once in the testing stage [42].

## 4. Experimental Results

### 4.1. Experiments

The learning models discussed in Section 3 were trained based on the CKD dataset, and the performance evaluation of each model was estimated using 10-foldcross-validation. During implementation, after setting all parameters, a confusion matrix was computed for building each model. This matrix provides four important measures [43]: true positive (TP), true negative (TN), false positive (FP), and false negative (FN), that are considered the basis for computing several other important measures: accuracy, precision, sensitivity, F-measure, specificity, and ROC/AUC.  Figure 3 shows the confusion matrix of the prediction models.

The performance of the models was evaluated using the following measures:

(i) Accuracy is the fraction of correctly classified CKD patients to the whole number of predicted patients [44]. (1) calculates the accuracy of the models.
  (1) $$\begin{array}{c} Accuracy=\frac{TP+TN}{TP+TN+FP+FN}\text{.} \end{array}$$
(ii) Precision is the fraction of accurately classified patients with CKD to those having CKD [37]. (2) calculates the precision of the models.
  (2) $$\begin{array}{c} Precision=\frac{TP}{TP+FP}\text{.} \end{array}$$
(iii) Sensitivity is the fraction of accurately classified CKD patients to the whole number in that class [37]. (3) calculates the sensitivity of the models.
  (3) $$\begin{array}{c} Sensitivity=\frac{TP}{TP+FN}\text{.} \end{array}$$
(iv) F-measure is the harmonic average of precision and sensitivity [45]. (1) calculates the F-measure of the models.
  (4) $$\begin{array}{c} F-measure=\frac{\left(2*precision*recall\right)}{precision+recall}\text{.} \end{array}$$

### 4.2. Results and Discussion

In the proposed models, KNN outperformed, and results compared to the existing prominent method are shown in Table 1.

Table 1 shows the overall reliability and efficacy of the proposed KNN method for early detection and diagnosis of CKD patients. Although KNN outperformed other methods, this study has tested the same dataset on other methods and reported the results in the following.  Table 2 shows the accuracies of each trained model computed based on (1).

As shown in Table 2, the performance of all prediction models is reasonable; KNN outperformed with 99.50% accuracy followed by SVM (99%) and bagging (98.50%).

Kappa values [46] are used to compare perceived accuracy with expected accuracy [47]. Kappa value higher than 0.75 is excellent [48]. In Table 2, the kappa values surpass the threshold and thus provide evidence of accurate models.

Moreover, the respective accuracies of the prediction models for detecting and diagnosing CKD were also estimated using other significant measures: precision, sensitivity, F-measure, specificity, and AUC score. These measures are computed based on the measures of the confusion matrix. First, recall or sensitivity is the amount of real positive values that are accurately labeled as positive, whereas precision is the predictive positive values or confidence of a model [49]. Likewise, the harmonic mean of sensitivity and recall is referred to as F-measure [50].  Table 3 shows the values of precision, sensitivity, F-measure, specificity, and AUC score for models trained in this study.

Furthermore, the models trained for detecting and diagnosing CKD were also examined using receiver operating characteristic (ROC) curve evaluation [51]. These curves are usually used in healthcare decision making and are greatly useful for creating classifiers and visualizing the trade-off between sensitivity and (1-specificity) [52] which is known as an efficacious measure of the intrinsic validity of a diagnostic test [53].  Figure 4 shows the ROC curves of all prediction models.

In ROC curves, the graphical comparison of two or more analytical tests can be performed at the same time in one graph, which is an advantage over individual values of precision and recall [53]. Furthermore, the classifier which provides a curve closer to the left upper corner shows better performance [37].  Figure 4 shows that the curves provided by the classifiers used in this study are almost on the left upper corner, providing evidence of the high performance of the trained models for detecting and diagnosing CKD.

The aforementioned tables and figures show that the models trained based on the CKD data are significantly reliable in terms of model accuracies, model performance, model sensitivities, F-measures, and the significantly reliable curves provided by the classifiers. This study has trained several models described above with an outcome of higher performance for all; therefore, they can be used as predictive models to help healthcare practitioners in detecting and diagnosing chronic kidney diseases and can also be an integral part of the CKD intervention decision-making process.

Moreover, due to the higher performance of the proposed models, they can be used as a decision support system for quick medical decisions in order to diagnose the CKD patients early based on the predominant features discussed in this study. Similarly, the feature selection process was applied in order to select the most relevant features for detecting and diagnosing CKD. Therefore, the soaring costs can be controlled by conducting fewer clinical tests and avoiding other identical tests, which may aid Third World survival.

The study employed different evaluation methods to examine the models, which increases the reliability of diagnosing the cases. In addition, the simplicity of the proposed method makes the implementation and deployment of such a system achievable.

## 5. Conclusions and Future Work

This study aims to develop prediction models for detecting and diagnosing CKD based on predominant features using machine learning techniques. In addition, to help reduce clinical expenses incurred by patients who are prescribed multiple identical tests, fewer mandatory tests sufficient to detect CKD can be performed instead. Several preprocessing steps have been applied to the dataset, such as missing value imputation, normalization, and feature selection. The processed dataset was trained using different prediction models such as KNN, SVM, RF, and bagging. The models' performance was estimated to show higher reliability and significance in terms of accuracy, sensitivity, F-measure, specificity, and AUC score. KNN outperformed the existing state-of-the-art methods used in the literature, showing the efficacy of the model to be used as a decision-making system for detecting and diagnosing CKD in the early stages.

Although the dataset contains all possible attributes that are enough to detect CKD at the early stage, there is a need for additional attributes that can aid in detecting CKD. In the future, the attributes such as GFR and eGFR which are also the main predictors for detecting CKD at the early stage could be added, and the performance of the trained models could be tested.

## Figures and Tables

**Figure 1:** Dataset description and values [22].

**Figure 2:** Dataset after feature selection.

**Figure 3:** Confusion matrix of all prediction models.

**Figure 4:** ROC curves of prediction models.

**Table 1:** Result comparison with existing methods with the similar dataset used in this study.

Study	Method	Accuracy (%)	Sensitivity (%)	Specificity (%)	AUC (%)	Precision (%)	F-measure (%)
[14]	RF	98.83	98.04	1.00	98.9	—	—

[13]	SVM	99.30	—	—	—	—	—

[8]	LR	99.24	100	—	—	98.82	—

[17]	XGB	99.00	98.8	99.33	99.9	99.5	99.1

[11]	MLP	98.10	98.97	96.77	99.50	97.97	98.4
	LR	98.10	98.97	96.77	99.4	97.97	98.4

Our method	KNN	99.50	99.20	98.70	99.60	100	99.60

**Table 2:** Accuracies and kappa values of prediction models.

S. no	Method	Accuracy (%)	Kappa value (%)
1	KNN	99.50	98.94
2	SVM	99.00	97.88
3	RF	98.75	97.32
4	Bagging	98.50	96.79

**Table 3:** Classification report of prediction models.

S. No	Method	Precision	Sensitivity	F-measure	Specificity	AUC
1	KNN	1.000	0.992	0.996	0.987	0.996
2	SVM	1.000	0.984	0.992	0.974	0.992
3	RF	0.984	0.996	0.990	0.993	0.998
4	Bagging	0.984	0.992	0.988	0.987	0.990

## Data Availability

The dataset used in this study was harvested from the publicly available UCI Machine Learning Repository [22].
